The article "Image Recognition of Pediatric Pneumonia Based on Fusion of Texture Features and Depth Features" was published in 2022. Journal: Comput Math Methods Med.

# Image Recognition of Pediatric Pneumonia Based on Fusion of Texture Features and Depth Features

**DOI:** 10.1155/2022/1973508

**Published:** 2022-08-26

**Authors:** Hao-Nan Wang, Li-Xin Zheng, Shu-Wan Pan, Tan Yan, Qiu-Ling Su

**Affiliations:** ^1^College of Engineering, Huaqiao University, Quanzhou 362021, China; ^2^The 910th Hospital of the Joint Support Force of the Chinese People's Liberation Army, Quanzhou 362008, China

## Abstract

Pneumonia is one of the diseases that seriously endangers human health, and it is also the leading cause of death of children under the age of five in China. The most commonly used imaging examination method for radiologists is mainly based on chest X-ray images. Still, imaging errors often result during imaging examinations due to objective factors such as visual fatigue and lack of experience. Therefore, this paper proposes a feature fusion model, FC-VGG, based on the fusion of texture features (local binary pattern LBP and directional gradient histogram HOG) and depth features. The model improves model performance by adding detailed information in texture features to the convolutional neural network while making the model more suitable for clinical use. We input the X-ray image with texture features into the modified VGG16 model, C-VGG, and then add the Add fusion method to C-VGG for feature fusion so that FC-VGG is obtained, so FC-VGG has texture features detailed information and abstract information of deep features. Through experiments, our model has achieved 92.19% accuracy in recognizing children's pneumonia images, 93.44% average precision, 92.19% average recall, and 92.81% average F1 coefficient, and the model performance exceeds existing deep learning models and traditional feature recognition algorithms.

## 1. Introduction

Pneumonia is one of the most common infectious diseases in clinical medicine. According to the World Health Organization, pneumonia is the leading cause of death among children under five. Moreover, more than 90% of children with childhood pneumonia are located in developing countries with limited medical resources [1, 2]. Therefore, an accurate and rapid diagnosis of pneumonia is essential in the treatment process. As the primary tool for the clinical diagnosis of pneumonia [3], a radiologist can diagnose based on a chest X-ray image. Still, the diagnosis requires the radiologist to have rich professional knowledge and clinical experience. At the same time, the doctor is also prone to misdiagnosis due to visual fatigue, background differences, and mental state differences [4].

With the increase in medical imaging data and the deepening of artificial intelligence research, artificial intelligence has also made significant breakthroughs in the medical field [5–9]. At the same time, deep learning also has an excellent performance in disease classification [10–12]. Deep learning methods have been clinically applied in areas such as aided diagnosis of lung nodules [13, 14] and aided diagnosis of breast cancer [15, 16]. However, there is still a big gap between the additional diagnosis model of pneumonia and its practical application in clinical medicine. Because various organs overlap, the lesion area is not prominent in the chest X-ray image. The lesion area has blurred boundary contours, different shapes and sizes, uneven density, etc. It is difficult for convolutional neural networks (CNNs) to extract deformations and features of chest X-ray lesions [17].

To overcome the problem of the lack of detailed information on the deep features of the above convolutional neural network, we use feature fusion technology to achieve information complementarity between traditional features and deep features [18]. At the same time, feature fusion technology also uses various kinds of information from medical images. Therefore, we propose a convolutional neural network model (FC-VGG) based on the fusion of texture features and depth features, modified on the VGG16 [19] network structure to make the model more suitable for auxiliary diagnosis of pneumonia. At the same time, to solve the problem of insufficient detailed information on deep features, we introduce a method of fusion of traditional features and deep features, which realizes feature layer fusion and makes the fused features more expressive than subfeatures. As a result, the FC-VGG model has stronger robustness and recognition performance for pneumonia images.

## 2. Related Work

In this section, we summarize the existing traditional feature pneumonia recognition methods, deep learning pneumonia recognition methods, and feature fusion pneumonia recognition methods.

In the field of pneumonia recognition, machine learning methods were mostly used in the early days [20–22]. This approach starts with image preprocessing, lung region segmentation, and other steps, followed by feature extraction and feature classification. Traditional image features have different features, such as texture, color, and shape. For the characteristic that chest X-ray images are grayscale images and contain a lot of texture information simultaneously, this paper uses texture feature extraction methods. Current texture feature extraction algorithms include local binary pattern (LBP), histogram of orientation gradient (HOG), and grayscale coevolution matrix (GLCM) [20, 23, 24]. The application of texture features is effective in pneumonia classification, so scholars usually use local texture features to represent pneumonia images [25]. In 2016, Pradeebha and Karpagavalli [26] used plain Bayes, decision tree, multilayer perceptron (MLP), and support vector machine (SVM) for classification and histogram of orientation gradient (HOG) feature for classification of pulmonary diseases. In 2021, Muhammad et al. [27] used various deep convolutional neural network (DCNN) migration learning techniques to extract useful features from chest X-ray images. Then, they trained and tested several machine learning classifiers on chest X-ray and CT image datasets. In 2021, Zhang [28] used machine learning methods to help radiologists make clinical decisions and screenings for COVID-19 lung imaging.

Nowadays, AI expands various applications in the medical field, such as disease classification [29, 30], medical image localization and detection [31, 32], and lesion region segmentation [33], and many deep learning-based models for lung disease identification are now available. In 2017, Rajpurkar et al. [4] proposed ChexNet, a 121-layer convolutional neural network model that not only detects 14 human diseases but also outperforms general radiologists in pneumonia classification. In 2020, Liang and Zheng [25] proposed a method that incorporates the idea of residuals and null convolution for childhood pneumonia recognition. They used the residual structure to overcome the overfitting and degradation problems of the deep model and used null convolution to overcome the problem of feature space information loss due to increasing model depth. In 2020, Yue et al. [34] used the dataset provided by Kaggle to train with each of the five mainstream network models, improved the network structure of MobileNet, and achieved higher accuracy. In 2020, Jain et al. [35] used six types of convolutional neural network models with various parameters to classify chest X-ray images into pneumonia and nonpneumonia categories. In 2020, Pérez [36] fine-tuned AlexNet by using 11312 chest X-ray images from six public databases to train the network model. In 2021, Narin et al. [37] used five pretrained convolutional neural network-based models (ResNet50, ResNet101, ResNet152, Inception V3, and Inception-ResNetV2) that can accurately detect COVID-19 using chest X-ray slices.

The purpose of feature-level fusion is to merge two or more features into one kind of new feature, and the expression capability of the fused features is superior to that of the original features. Also, the result of feature fusion can contain richer information about the dataset [38]. In 2019, Xinyu and Zhang [39] proposed a deep convolutional neural network- (DCNN-) based algorithm for pneumonia image recognition. An Inception V3 network model trained using the ImageNet dataset is used to extract features. Then, a feature fusion layer is added to fuse the features, and a random forest classifier is used for classification and prediction. In 2019, Han et al. [40] extracted features from convolutional neural networks (CNN) and classical methods (HOG and LBP). Then, the CNN-HOG features are compressed by the principal component analysis (PCA) algorithm and combined with the LBP features to obtain the fusion features. Finally, the fused features train the SVM model to improve the classification performance.

Most of the scholars in the articles mentioned above have made good progress in their research areas and contributed to the development of artificial intelligence in the medical field. Still, the studies mentioned above also have some problems.

1. Machine learning approaches using traditional features all perform traditional feature extraction and then classify based on the features, but this ignores the connection of deep information in images and has poor performance in the face of nonlinear decision problems like pneumonia recognition
2. Using the deep learning approach, abstract features are obtained from the original image for classification. Still, this approach is not sensitive enough to the various overlapping organs and lesion regions in chest X-ray images, and their depth features usually lack spatial and detailed information. This also leads to a limitation of classification accuracy. Moreover, lesion regions have fuzzy boundary contours, different shape sizes, uneven densities, etc., and it is difficult for convolutional neural networks (CNNs) to extract deformations and features of chest X-ray lesions
3. Using the feature fusion approach of deep learning and machine learning, the complementary information of abstract features of deep learning and detailed features of machine learning can be realized. However, this fusion approach requires different traditional features, deep learning network models, and fusion methods to be selected for different recognition tasks. Otherwise, feature fusion will not only be affected by the information of subfeatures but also add more parameters and consume more computational resources. In contrast, the model performance will be affected

The main contributions of this paper are summarized as follows: (1) we produced a database containing 13040 chest X-ray images of children aged 2 to 14 years. (2) We improved the VGG16 model (C-VGG) for the pneumonia classification task, which reduces the number of parameters and overfitting phenomenon compared to VGG16. (3) We propose a feature fusion model based on the fusion of texture features with depth features, FC-VGG. The texture features in the model contain LBP and HOG features. Then, we input the texture feature images into C-VGG and then fuse the features by Add fusion. Thus, the model achieves complementary texture feature detail capture capability and depth feature abstraction capability. Meanwhile, the robustness and recognition performance of the FC-VGG model for pneumonia images are improved under the validation of several evaluation criteria. Meanwhile, the robustness and recognition performance of the FC-VGG model for pneumonia images are improved under the validation of several evaluation criteria.

## 3. Datasets and Methods

### 3.1. Data Sources and Data Collection

This experiment's pediatric pneumonia imaging dataset included a chest X-ray database of pediatric patients aged 1-5 years (ChestXRay2017) and a chest X-ray database of pediatric patients aged 2-14 years. The data were obtained from Guangzhou Women's and Children's Medical Center and a hospital in Quanzhou, respectively. Pediatric pneumonia patients and healthy kids from Guangzhou Women and Children's Medical Center's chest X-ray images are referred to as GP-Xray and GN-Xray, respectively, and healthy kids from a hospital in Quanzhou's chest X-ray images are referred to as QP-Xray and QN-Xray, respectively.  Figure 1 shows a schematic diagram of the different types of chest X-rays in the database.

Since the image sizes of the datasets in this paper vary, we need to perform image preprocessing. We finally added a total of 13,040 chest X-ray images of children to the experiments, and we collected the data from pediatric patients aged 1-14 years. Meanwhile, we used the K-fold cross-validation method for data assignment during training, which can ensure the random assignment of experimental data and the stability of the model. The amount of data in each category is shown in Table 1:

#### 3.1.1. Data Preprocessing Process

Many of the images in the acquired pediatric chest film dataset contain large areas of useless background information, and each image is of a different size. These often cause interference and recognition difficulties. Therefore, we subjected the children's chest X-ray image dataset to a preprocessing operation by first cropping the original images, then normalizing them by the maximum and minimum value methods, and finally scaling the image size to 224∗224 pixels in equal proportion.

### 3.2. Texture Feature Extraction

#### 3.2.1. Local Binary Pattern (LBP)

It is rapid, computationally light, illumination-insensitive, and rotationally undistorted, making LPB one of the best methods for defining texture features currently available. The original LBP operator compares the center of each pixel point with the gray values of the eight pixels around it, using the gray value of each pixel point in the image as the threshold value. One of the threshold values for the gray value of the adjacent pixel points is exceeded; otherwise, it is 0. The comparison is made in a certain order, and an 8-bit binary number is obtained, and this binary number is used as the LBP value for the pixel point. The LBP texture feature extraction process is shown in Figure 2.

The specific formula of the LBP algorithm is

(1) $$\begin{array}{c} {\text{LBP}}_{\left({\text{x}}_{\text{c}},y_{c}\right)}=\overset{i=7}{\underset{i=0}{\sum }}2^{i}s\left(q_{p}-q_{c}\right), \end{array}$$

(2) $$\begin{array}{c} s\left(g_{p}-g_{c}\right)=\left\{\begin{array}{cc} 1, & \left(g_{p}-g_{c}\right)\geq 0,\\ 0, & \left(g_{p}-g_{c}\right)<0, \end{array}\right. \end{array}$$

where *q*_*c*_ is the gray value of the center pixel point, *P* is the pixels point around the center pixel, *q*_*p*_ is the gray value of the *P* pixel point, and *s* denotes a symbolic function. Then, we transform the LBP values into grayscale images, i.e., images with LBP texture features.

#### 3.2.2. Oriented Gradient Matrix (HOG)

The directional gradient matrix method (HOG) is one of the most commonly used texture feature extraction methods today, and it is widely used for object classification and pedestrian recognition because it handles grayscale images better than color images. The basic principle of HOG is to use gradient information to describe the edges of an image and then characterize the local image using the magnitude of the gradient. The six steps of the HOG algorithm are the image grayscale HOG feature extraction process (shown in Figure 3).

The main calculation formula of the HOG algorithm is

(3) $$\begin{array}{c} \left\{\begin{array}{c} F_{x}=H\left(x+1,y\right)-H\left(x-1,y\right),\\ F_{y}=H\left(x,y+1\right)-H\left(x,y-1\right), \end{array}\right. \end{array}$$

(4) $$\begin{array}{c} G\left(x,y\right)=\sqrt{F_{x}^{2}+F_{y}^{2}}, \end{array}$$

(5) $$\begin{array}{c} \alpha \left(x,y\right)=\tan^{-1}\frac{F_{x}}{F_{y}}, \end{array}$$

where *F*_*x*_ and *F*_*y*_ are the gradient values of the pixel (*x*, *y*) in the image in horizontal and vertical directions, respectively, *H*_(*x*, *y*)_ is the gray value of the pixel in the image, *G*(*x*, *y*) is the mode length size of the gradient of the pixel point, and *α*(*x*, *y*) is the direction of the pixel point. After calculating the gradient information, we must additionally count the gradient histogram of each cell in various directions to create the descriptor of each cell. Next, we must connect all the cells to create the HOG feature matrix, which we must convert into a grayscale image.

### 3.3. Feature Fusion

There are roughly two types of feature fusion: early fusion and late fusion. Early fusion is to fuse the features of multiple layers first and then train the predictor on the fused features. Late fusion is to make predictions before the final fusion is completed and eventually fuse multiple predictions. We adopt the early fusion strategy since late fusion cannot solve the fundamental problem of insufficient feature information. Early fusion also contains various fusion methods such as Concat and Add. In this paper, we adopt the Add fusion method, which increases the amount of information under each dimension of the feature vector describing the image. At the same time, the dimensionality remains unchanged, and the computation of the Add method is much smaller than that of the Concat method. Finally, the texture and depth features are fused into a composite feature vector. The specific calculation formula of the Add fusion method is as follows:

(6) $$\begin{array}{c} Z_{\text{add}}=\overset{c}{\underset{i=1}{\sum }}\left(X_{i}+Y_{i}\right)*K_{i}, \end{array}$$

where *K*_*i*_ represents the weighted vector, *X*_*i*_ and *Y*_*i*_ is a vector of the two input channels, ∗ stands for convolution, and *Z*_add_ represents the fusion feature vector. The main purpose of Add fusion is to add up the corresponding feature maps in the two channels to achieve feature complementarity.

### 3.4. FC-VGG Model

The model proposed in this paper is designed to assist radiologists in the fast and accurate diagnosis of pneumonia images in children. For the image characteristics of various organs overlapping each other and lesion regions not prominent in chest X-ray images, this paper adopts a deep learning-based method that incorporates texture features and depth features to enrich the deep learning model's features. In this study, the chest X-ray pictures with texture features after feature extraction are input into the deep learning model. First, the LBP approach with grayscale invariance and the HOG method with direction invariance are utilized for texture feature extraction. In this study, the basic network is the VGG16, which mostly replaces large convolutional kernels with numerous small convolutional kernels. The nonlinear capacity of the network can be efficiently increased, while the number of network parameters is decreased by superimposing multiple tiny convolutional kernels. In addition, we remove the first fully connected layer (Fc) of the VGG16 model to reduce the large parameters, add the dropout layer to the second and third Fc layers of the VGG16 model in order to reduce the overfitting phenomenon, and change the output channels of the last Fc layer of the VGG16 model to 2 in order to meet the binary classificatory requirements. Then, the input of texture feature (with HOG and LBP features, respectively) images is added to C-VGG, and feature fusion is performed after the pooling layer in the model. The texture features are fused with the depth features by Add fusion of early fusion to form the fused feature vector, and then, the fused feature vector is trained, from which we obtain the FC-VGG model. A detailed model schematic (shown in Figure 4) is finally achieved to recognize and classify childhood pneumonia images.

## 4. Experiments and Analysis

### 4.1. Experimental Environment and Training Parameters

The computer configuration for this experiment is as follows: CPU is Intel(R) Xeon(R) Gold 5118; GPU is NVIDIA TITAN XP; video memory is 12 G; memory is 128 G; computer OS is 64-bit Linux-4.15; learning rate is 0.0001; epochs are set to 50; batch is set to 64; data allocation is done by 5-fold cross-validation method. Meanwhile, all experiments in this paper use the above equipment and parameters to ensure the same experimental conditions.

### 4.2. Evaluation Indicators

In multiclassification models, accuracy, precision, and recall are the main evaluation metrics to measure whether the algorithmic model is correct. However, in some cases, there is a conflict between recall and accuracy calculation methods. We introduce a common, comprehensive evaluation metric, F-measure, and a weighted sum of accuracy and recall, and the higher the *F*-value, the better the model performance. Each of the following evaluation metrics has its formula:

(7) $$\begin{array}{c} \text{Accuarcy}=\frac{\left(\text{TP}+\text{TN}\right)}{\text{TP}+\text{TN}+\text{FP}+\text{FN}}, \end{array}$$

(8) $$\begin{array}{c} \text{Precision}=\frac{\text{TP}}{\text{TP}+\text{FP}}, \end{array}$$

(9) $$\begin{array}{c} \text{Recall}=\frac{\text{TP}}{\text{TP}+\text{FN}}, \end{array}$$

(10) $$\begin{array}{c} F1=\frac{2\times \text{Precision}\times \text{Recall}}{\text{Precision}+\text{Recall}}, \end{array}$$

where TP is a true positive, indicating that the model predicts true and the actual result is also true; FP is a false positive, indicating that the model predicts true and the actual result is false; TN is a true negative, indicating that the model predicts false and the actual result is also false; and FN is a false negative, indicating that the model predicts false and the actual result is true.

### 4.3. Parameter Optimization Experiment

#### 4.3.1. LBP Algorithm Selection

There are also many variants of LBP algorithms, such as Uniform-LBP, Var-LBP, and Ror-LBP. Different LBP algorithms change their coding patterns to achieve different texture feature requirements. Therefore, different feature extraction algorithms have their advantages. Therefore, we will select the most suitable algorithm for this paper model by comparing several LBP algorithms. The experimental results and various indexes are shown in Table 2.

As shown in Table 2, after FC-VGG model training, the model in this paper obtained the best results when Var-LBP was used, and its values of Accuracy, Aver-Precision, Aver-Recall, and Aver-F1 score were the best among the various LBP algorithms, and the accuracy rate reached 84.23%. The Var-LBP algorithm also introduces local variance information, which allows the model to have a faster convergence speed.

#### 4.3.2. Cell Size Selection of HOG Algorithm

The HOG algorithm is to divide the image into multiple cells and then performs local feature extraction. Hence, the information in the HOG features depends on the cell size selection. Therefore, in this paper, the best cell size is obtained by FC-VGG model training, the experimental range is taken between [2,32], and the specific experimental results and various indexes are shown in Table 3.

As shown in Table 3, after the FC-VGG model training, the evaluation indexes show a decreasing trend when the cell size changes from small to large, and the best performance is achieved when the cell size takes the value of 2∗2, with an accuracy rate of 92.66%. The experimental results show that the cell size of HOG features will determine the model performance, and choosing the best cell size will positively affect the model classification performance.

#### 4.3.3. Selection of Fusion Positions in FC-VGG

The feature fusion method used in this paper will make the number of parameters of the network model too much. Therefore, we use the VGG16 model as the base network and modify the model to obtain C-VGG, which can reduce the parameters of the convolutional layer and, at the same time, has superior feature learning ability and detailed information capture. Therefore, FC-VGG can be divided into six positions, which are as follows: input, between the first convolution layer and the first maxpool layer (block 1), between the third convolution layer and the second maxpool layer (block 2), the fifth convolution layer and the third maxpool layer (block 3), between the eighth convolution layer and the fourth maxpool layer (block 4), and between the eleventh convolution layer and the fifth maxpool layer (block 5). The fusion in different positions of FC-VGG will determine the performance, the number of parameters, and the training speed of the model, so this paper conducts experiments for the fusion positions. The specific experimental results and the metrics are shown in Table 4.

The experimental results indicate that fusion at different block positions will have an impact on the model performance. As shown in Table 4, after training the FC-VGG model, this paper achieves the best performance after fusing traditional features between the fifth convolution layer and the third maxpool layer of FC-VGG (block 3).

### 4.4. Experimental Results

The best results of the FC-VGG model were obtained using the Var-LBP algorithm by optimizing the training of the above model parameters. We took cell size as 2∗2, the fusion position was block 3, and the overall recognition accuracy of this model for childhood pneumonia images was as high as 93.92%, the average accuracy reached 93.44%, and the average recall reached 92.19%. To better distinguish the strengths and weaknesses of this model, we will also compare the model in this paper experimentally with other known models.

### 4.5. Comparative Experiment

Since FC-VGG is a fusion model of traditional texture features and depth features, the comparison experiments mainly consist of current models compared with machine learning method models and deep learning models that have been successfully applied to childhood pneumonia at this stage in the same environment. With the same dataset, Table 5 includes the performance of machine learning models of LBP and HOG, VGG16, MobileNet, Inception V3, ChexNet [4], and FC-VGG.

From each evaluation index, we can see that the FC-VGG model in this paper achieves very good results. Our proposed method is 6.87% higher than the optimal MobileNet model in terms of accuracy, 5.39% higher than the optimal ChexNet model in terms of precision, 6.87% higher than the optimal MobileNet model in terms of recall, 8.13% higher than the optimal *F*1 value, and 8.13% higher than that of the optimal HOG+SVM model. Combined with the optimal selection of parameters in the previous paper, we adopted the Var-LBP feature extraction algorithm for the characteristics of pneumonia X-ray images and limited the cell sizes of HOG to 2∗2, then extracted the texture features that are helpful for pneumonia recognition, and then chose to fuse them at the position of block 3 in FC-VGG, so that the fused features have the detail information of texture features and the abstract information of depth features. The Add fusion method can keep the feature dimension constant while increasing the amount of information in the image feature vector. The results indicate that the model performance of FC-VGG is superior to the machine learning models of LBP and HOG because the deep learning method used in FC-VGG can obtain deep information directly from the image, and compared with deep learning models such as VGG16, FC-VGG can extract shallow texture features of the image and has more power to resolve the image. The model's performance in this paper is experimentally proven effective and has improved in all aspects compared to the ChexNet model for pneumonia-assisted diagnosis.

### 4.6. Discussion

Experimentally, it is proved that the convolutional neural network model with texture features fused with depth features proposed by our proposed FC-VGG model can effectively classify the X-ray images of childhood pneumonia. However, this paper has some shortcomings, which will be the goal of future research. Firstly, the parameter size of the C-VGG structure proposed in this paper is too large. For a real-time task like pneumonia recognition, we would like to achieve its parameter size reduction while keeping the accuracy rate constant. We can also optimize the C-VGG model structure by using model compression to reduce the number of parameters. Secondly, we can improve the fusion method in FC-VGG. We can use PCA (principal component analysis), DCA (decision curve analysis), and other fusion methods to downscale the features so that the features become linearly irrelevant to make feature fusion easier and to improve the model's computational speed. Finally, we can start from the data image, image segmentation for the characteristics of child pneumonia X-ray images, while adding deep learning adversarial example image generation method, which can reduce the interference features of the image. In contrast, the adversarial sample makes the model can still be satisfied when dealing with abnormal image input.

## 5. Conclusion

To help radiologists make a more rapid and accurate diagnosis of pediatric pneumonia. In this paper, we propose a classification model based on the fusion of texture features (LBP and HOG) and depth features for pneumonia image recognition in children, FC-VGG. This model improves the network structure of VGG16, reduces the number of parameters and overfitting phenomenon of the model, and makes it have better performance results for the binary classification task of pneumonia image recognition. Meanwhile, two texture feature methods are used in this paper to collect richer texture information, and the various parameters of the methods are trained. Finally, this paper uses Add fusion to incorporate texture features of pneumonia images into the model while ensuring the integrity of texture information, so the fused features of the model are rich in texture information and abstract depth features of pneumonia images. In this paper, we use the K-fold cross-validation method to assign data to achieve the classification of pneumonia images in children by training the FC-VGG model. The comparison of experiments and evaluation metrics in this paper shows that our model greatly improves recognition accuracy compared with traditional machine learning algorithms and deep learning algorithm models, and its prediction accuracy can reach 92.19%. The experiments prove that the FC-VGG model proposed in this paper can effectively recognize and classify children's pneumonia images. Therefore, the FC-VGG model can solve the problems of radiologists' visual fatigue and inexperience, leading to diagnostic errors. At the same time, it can effectively save manpower and medical resources and improve work efficiency. Finally, we hope that the model method in this paper can be further applied in clinical practice to provide radiologists with diagnostic criteria for childhood pneumonia.

## Figures and Tables

**Figure 1:** (a and c) The medical images of the pneumonia chest X-ray in two hospitals, respectively, and (b and d) the medical images of the chest X-ray with confirmed pneumonia.

**Figure 2:** Schematic diagram of LBP feature extraction.

**Figure 3:** Schematic diagram of HOG feature extraction.

**Figure 4:** Schematic diagram of FC-VGG model.

**Table 1:** Various data volumes.

Data sources and types	Total data	Training set	Test set
GP-Xray	4273	3420	853
GN-Xray	1583	1110	473
QP-Xray	5127	4102	1025
QN-Xray	2057	1646	411
Total	13040	10278	2762

**Table 2:** Model performance using different LBP algorithms.

LBP algorithm	Accuracy (%)	Precision (%)	Recall (%)	*F*1 score (%)
Default-LBP	78.53	79.02	80.23	79.62
Nri-uniform-LBP	63.64	76.06	63.64	69.29
Uniform-LBP	60.41	56.29	60.41	58.27
Ror-LBP	66.59	73.17	66.59	69.72
Var-LBP	84.23	84.83	84.23	84.52
Circle-LBP	35.62	38.14	35.62	36.83

**Table 3:** Model performance using different cell sizes.

Cell size	Accuracy (%)	Precision (%)	Recall (%)	*F*1 score (%)
2∗2	92.66	91.09	91.94	91.51
4∗4	84.91	86.37	84.91	85.63
8∗8	82.73	84.89	82.73	83.79
16∗16	81.29	82.84	81.29	82.05
32∗32	81.14	82.46	81.14	81.79

**Table 4:** Performance of postfusion of each block in FC-VGG.

Model	Accuracy (%)	Precision (%)	Recall (%)	*F*1 score (%)
Input	92.06	91.52	91.45	91.48
Block 1	88.33	89.96	82.70	86.17
Block 2	90.78	88.98	89.60	89.28
Block 3	93.92	93.44	92.19	92.81
Block 4	92.42	92.74	92.36	92.54
Block 5	88.61	91.45	82.25	86.60

**Table 5:** Performance of each model.

Model	Accuracy (%)	Precision (%)	Recall (%)	*F*1 score (%)
LBP+SVM	77.59	76.18	77.59	76.87
HOG+SVM	83.49	85.91	83.49	84.68
VGG16	72.01	53.53	72.01	61.40
MobileNet	85.32	82.68	85.32	83.97
Inception V3	67.54	68.88	67.54	68.20
ChexNet	79.80	88.05	79.80	83.72
Ours	92.19	93.44	92.19	92.81

## Data Availability

Data is available on request from the authors due to privacy/ethical restrictions.
